# Assessing the management student's entrepreneurial intentions: Role of entrepreneurship education and technology transfer

**DOI:** 10.3389/fpsyg.2022.953324

**Published:** 2022-08-08

**Authors:** Zihan Wang, Geovanny Genaro Reivan Ortiz

**Affiliations:** ^1^School of Education, The University of Sheffield, Sheffield, United Kingdom; ^2^Henan Association of Cultural History, Zhengzhou, China; ^3^Laboratory of Basic Psychology, Behavioral Analysis and Programmatic Development PAD-LAB, Catholic University of Cuenca, Cuenca, Ecuador

**Keywords:** entrepreneurial intentions, technology transfer, entrepreneurial training, entrepreneurship education, partial least squares

## Abstract

Entrepreneurship education is considered as an important way to influence the competitiveness of any country or industry. Therefore, entrepreneurship education provides opportunities to progress to a more competitive educational environment. This paper examines the impact of students' entrepreneurship education in China on their entrepreneurial intentions. Perceived entrepreneurial capacity, education in entrepreneurship, and attitudes toward entrepreneurship are all factors in the model developed to predict entrepreneurial intention. Structured equation modeling (SEM) is being used to test 98 management students from various universities in China. The findings show that there is statistically significant and positive relationship among entrepreneurship learning, entrepreneurial attitude, entrepreneurship education, and management students' entrepreneurial intention. Perceived behavioral control and perceive social rule significantly improve management students' entrepreneurial intention. Moreover, technology transfer correlates statistically with students' entrepreneurial intentions. Thus, universities are being encouraged to offer entrepreneurial training modules to increase their students' entrepreneurial intent.

## Introduction

Formal education produces entrepreneurs with a greater impact on national wealth than self-made entrepreneurs (Huang et al., 2021). Entrepreneurship programs and courses have mushroomed in colleges and universities all over the world due to this widely held belief (Mukonza, 2016; Huang et al., 2021). However, there is still much to learn about education and entrepreneurship training (Wang et al., 2020; Anshika and Mallik, 2021; Purwandari et al., 2022), as research in this area is still in its infancy. It is common knowledge that entrepreneurship is the process of conceptualizing, creating and running a new business, usually as a small business such as a start-up firm, to provide a good or service to the public (Cheng and Wang, 2022; He et al., 2022). Because of its importance and specificity and a large number of concerned parties, entrepreneurship is becoming increasingly popular as a means of contributing to financial growth by providing a wide range of services and products that are beneficial to all industries; alongside the new services, it will also result in an enormous increase in employment and products they present in the marketplace (Mukonza, 2016; Stanislavská et al., 2020; Ramírez-Montoya et al., 2021). With the emergence of a knowledge-based economy, a high level of financial performance necessitates the use of new technology and innovation. Technology and business incubators are widely used in this direction and are known to generate new technology commercialization tools and initiative expansion (Ratten and Jones, 2021; Gavriluţǎ et al., 2022).

Several universities worldwide have developed training and research programs on sustainable entrepreneurship in a significant manner to build sustainable social order (Khan, 2019; Jin, 2022). Educators frequently deliver sustainable entrepreneurship education by integrating relevant subjects by educators (Butkouskaya et al., 2020). Aside from improving their skills, graduates of sustainable entrepreneurship training gain new contacts that will aid them in their future careers (Purwandari et al., 2022). Students, for example, access to various networks is possible by affiliating themselves with academic institutions. Young people's desire to learn about sustainable business practices is growing (Havidz et al., 2018). For example, Morgan and Trinh (2019) points out that in Hong Kong, there is a growing demand for sustainable competitions, entrepreneurship courses, and extracurricular activities. Moreover, entrepreneurial talent can be harnessed, and new businesses can grow faster if the business incubator can efficiently connect people, knowledge, resources, and technology.

Using China's higher education institutions as a case study, this paper examines how they can help students and the wider community by providing high-quality business education to prepare them to start their businesses (Sun and Razzaq, 2022). A global trend in educational strategy includes a statement on entrepreneurship in business faculties (Cook et al., 2014). Higher education, especially at the college level, is critical. In the meantime, a heated debate has raged in the region since the turn of the 21st century over the role education should play in creating a society that relies heavily on “entrepreneurship.” There is no doubt that entrepreneurship is a top priority for the government and businesses after reviewing the current education program (Yoon and Zhang, 2018). According to prior research, universities play a significant role in business, demonstrating the educational system's importance for entrepreneurial learning (Kasilingam, 2020a).

In recent years, entrepreneurship research has piqued the curiosity of academics, practitioners, and public officials alike (Kozup and Hogarth, 2008; Lusardi and Mitchell, 2013; Shaouf et al., 2016). It is widely accepted that entrepreneurship education and training are strong tactical tools for regional growth. This study aims to investigate the management student's entrepreneurial intentions under the role of entrepreneurship education and technology transfer. The study contributes in the existing literature as fallows: First, this paper gives a theoretical foundation for the variables under consideration by reviewing previous studies conducted worldwide. Second, this paper provides a theoretical framework with hypotheses to better understand the relationships between variables in the study. According to Bolaños et al. (2022), only a few studies have been done within developing countries on entrepreneurship schooling or education; however, these studies have focused on the influence of entrepreneurship education on definite fields (Edwards et al., 1998; Kim et al., 2021). Especially in the China context, as far as the authors were aware, there had never been a study on this subject. Consequently, this study aims to analyze the impact of the supply of entrepreneurial ventures to the business market by public higher education in China (China public institutions, JPIs). The influence of business incubators on students' ability to develop new venture ideas that set new business trends is also being investigated.

First, we conduct a literature analysis on the subject matter under consideration. After that, we'll work on showing students what it means to be an entrepreneur. In addition, the approach used to gather the data will be made public. Finally, the subject of this article will present the most important findings, enlightening and concluding on the assistance, and the boundaries of this effort and outlooks for the future.

## Literature review and hypotheses development

Researchers, practitioners, and politicians are keenly interested in the determinants of entrepreneurial intention. This topic still requires further exploration (Burton-Jones and Hubona, 2006; Starr and Starr, 2021); further research is therefore required. Various factors likely influence young people's entrepreneurial level, but the exact nature of those influences varies from researcher to the next. Shapiro's model of the entrepreneurial event and Ajzen's planned behavior model are the two main reference models that empirical research has used to examine this issue. Thus, we use these two models in an integrated approach to recognizing the factors that students' entrepreneurial aspirations should be supported (Lee and Brahmasrene, 2013; Alsabawy et al., 2016; Kasilingam, 2020b). Theory of planned behavior (TPB) had only three gages before personal intention: boldness toward the concerning behavior, perception of perceived behavioral control (TPB-BPC), and communal norms (Figure 1). A person's actions are directly influenced by their level of intent (Field, 2020; Stanislavská et al., 2020; Ambalov, 2021). According to Shen et al. (2016), an individual's attitude measures how much they value certain behaviors. Individual behavior is influenced by social norms (such as the views of one's parents and other relatives). It is thus possible to define behavioral control by referring to the difficulties that an individual must overcome in a given behavior, dependent on the accessibility of resources (George et al., 2012). If you ask someone about their intention, they will say, “how hard they are willing to try, how much effort they are planning to exert (Klapper et al., 2013). Experts are unanimous in their belief that TPB can be a powerful tool in studying entrepreneurial intention (Alsabawy et al., 2016).

**Figure 1:** A model for predicting the entrepreneurial intentions of management students.

### Students' entrepreneurial intentions

Many researchers around the world are interested in studying the determinants of students' entrepreneurial intentions (Razzaq et al., 2020; Khan et al., 2021; Fang et al., 2022). Indeed, a number of studies have shown that exposure to entrepreneurship education can significantly influence a person's entrepreneurial aspirations. Although there is a wide range of incubators for small businesses, they all have the same goal: to aid in establishing, expanding, and maintaining new entrepreneurial ventures. As well as providing experienced administrative help, laboratory space or low-cost office, management services, and access to a network of specialists such as investors, auditors and lawyers, these kinds of organizations share specific features. This kind of support enables the entrepreneur to focus on product development and advertising policies rather than managerial and functional problems (Hoskisson et al., 2013; Calcagno and Monticone, 2015; Juliansyah, 2019).

Investing in human capital is a way for China, a rising country with inadequate capital, to manage its situation (Sun et al., 2022a). The problems in neighboring countries have recently had a negative impact on the economy, which has resulted in a decrease in GDP and an increase in borrowing to compensate (Vasic et al., 2019). It follows those entrepreneurial ventures, which are based on creative and novel ideas rather than financial capital, are needed as a tool for fiscal growth (Jiang et al., 2021; Osuret et al., 2021). In several developed countries, business incubators have proven to be an effective tool for combating unemployment, spreading economies, and creating wealth. An entrepreneurial culture can be fostered on both the micro and macro scales by providing timely assistance and funding to new businesses in need of assistance and funding (Chen et al., 2020). In addition, earlier studies have shown that the graduates of business incubators have higher levels of endurance and prosperity (Zhang et al., 2022). Consequently, incubators may benefit a wide range of companies. Despite this, they are frequently set up to assist technology-based companies by providing a wide range of start-up businesses. The incubator aims to accelerate technology marketing by bridging the gap between human capital, technical expertise, and financial resources (Das et al., 2019).

### Education and entrepreneurial learning

People are seen as dynamic suppliers and tools for improving the conditions surrounding their lives in the Social Cognitive Theory (SCT) (Lu et al., 2016). On the other hand, goals can be pursued if individuals believe their activities and abilities can achieve the desired consequences (Hsu et al., 2021). Learning about entrepreneurship helps students improve and enhance their cognitive abilities, constantly modify their activities and ideas, and create consistent, meaningful, and focused entrepreneurship (Havidz et al., 2018; Sun et al., 2022b). Entrepreneurship education has been used in other contexts to emphasize the importance of analyzing the influence of various variables such as risk-taking, proactiveness, self-efficiency, and demographic on entrepreneurial intentions even though demographic variables are still stifling (Abdullah et al., 2016).

Our work is based on the concept of “govern-mentality” established by Ma and Bennett (2021) in our research (Doha et al., 2019; Wang et al., 2021). There must be an understanding of how “govern-mentality” relates to educational issues, particularly the training of entrepreneurs (Doha et al., 2019; Sharma and Aggarwal, 2019; Zhang and Ramse, 2021). Rather than the traditional meaning of the word “government,” this phrase conceptually combines the words “govern” and “mentality,” reflecting a broader range of ways to rule (Juliansyah Noor, 2019). Because of this, the techniques used by powers and individuals differ greatly. In contrast to the power's methods of defining people's behavior and assigning them to specific domination goals, the methods of individuals refer to the formation of individuals' methods of self-construction of citizenship. Subsequently, these methods allow people to perform a precise number of processes on their bodies, behavior, politics and way of being through their methods or with the assistance of others (Tiep et al., 2021).

Since we live in a rapidly-shifting world, the most pressing issue is how to raise citizens who are able to adjust to new situations quickly and effectively. Persons with high levels of consciousness and responsibility, who can take control of their own lives (including work, family, education and other activities) based on their principles, situations and desires, are essential to building this society. Individuals who are shaping the next generation and must be ready for such a rapidly shifting environment must be highly motivated, skilled, and knowledgeable, as well as able to take the initiative to further their advancement and the wellbeing of the society in which they reside (Castro et al., 2022). Collective efforts from the governments are needed to educate individuals to be more attentive to the concept of globalization and the quick change of environment in addition to the self-skills that some people have already developed (Baah et al., 2021), mainly in the business field (Tajvidi et al., 2020).

In today's world, education is no longer a question of what students learn in school and university; rather, it is a sign of the ultimate education that permeates all aspects of society (Dashti et al., 2019). As a result, an increasing number of policymakers and scholars in the education and business fields are focusing on this topic and tying financial development and growth to entrepreneurship education or schooling (Shaouf et al., 2016; Ambalov, 2021). Furthermore, public education systems play an important role in encouraging students to become entrepreneurs by providing entrepreneurship programs and courses (Choi and Mai, 2018; Havidz et al., 2018; Haldorai et al., 2022).

Indeed, incubation has been suggested to encourage entrepreneurial activity and start-ups, leading to new strategy incentives. Real entrepreneurship, it has been asserted, has its origins in the incubation process. Graduates are also able to start their businesses outside of the nurturing buildings, which has a positive result on the entrepreneurial mindset and the establishment of a strong connection between R and D sectors, business and universities, as well as a construction that allows access to fiscal markets (Ashraf et al., 2021a). This emphasis on education has necessitated the creation of new knowledge. As a result, aptitudes and services regarding start-up businesses, leadership, and problem-solving in education courses and programs (Das et al., 2019; Morgan and Trinh, 2019).

### Business incubators and entrepreneurship ventures

Incubators aid an increase in the number of start-up companies by providing assistance and backup services (Cook et al., 2014). In addition, business incubators are seen as a critical component of economic development plans at the local and state levels (Anshika and Mallik, 2021). Failure in this context is associated with the absence of complete business support, primarily service-based customers rather than manufacturing-based, and incubation grounds that are poorly constructed or professional. These factors impact the total amount of money that the incubator helps to generate (Yu et al., 2005).

In several developed countries, business incubators have proven to be an effective tool for combating unemployment, spreading economies, and creating wealth. An entrepreneurial culture can be fostered on both the micro and macro scales by providing timely assistance and funding to new businesses in need of assistance and funding (Jurca, 2008; Aboramadan and Karatepe, 2021). In addition, earlier studies have shown that the graduates of business incubators have higher levels of endurance and prosperity (Shaouf et al., 2016). Since they can help a wide range of businesses, incubators are often created to aid technology-based businesses by providing various resources and assistance to start-ups. The incubator aims to accelerate technology marketing by bridging the gap between human capital, technical expertise, and financial resources (Kim et al., 2021).

Government funding usually establishes business incubators to create jobs, revitalize the economy, or promote new ideas (Kim et al., 2021). Entrepreneurial societies and organizations benefit from incubators, which act as a catalyst for developing corporate business support systems, such as financial institutes, educational institutions, large corporations and professional organizations such as the government. This means that an incubator located in a location with a higher concentration of similar and diverse businesses will have an easier time gaining access to the capital needed by new entrepreneurial ventures. As many businesses are located in the same geographic area, new businesses can access a wider range of technical and scientific data unavailable in regions where businesses are spread out or in smaller numbers (Wang et al., 2011).

Supervisory services, endowment services, particular customer service and personal services provided by technological business incubators in China have recently been found to play an important role in supporting small businesses and enhancing their marketing abilities (Lu et al., 2010). As a result, various new forms of support for budding entrepreneurs are emerging. Unlike in the past, these new forms of support have a much greater and more widespread impact on the community than common knowledge-based methods. Entrepreneurship can be boosted through start-up incubation (Cui et al., 2018). Aside from knowledge transfer, incubators can help businesses or individuals by providing services and resources. In turn, this will aid in forming links between businesses and entrepreneurs (Juliansyah, 2019). As a result, incubators ensure the stability of businesses, financial development, and long-term venture survival (Singhal et al., 2019). Incubators regularly produce constructive businesses (Gluch et al., 2009; Jové-Llopis and Segarra-Blasco, 2018). According to previous research, the author concluded that:

**H1: Entrepreneurial ventures attitude are directly and positively associated with Students' entrepreneurial intentions**

### Entrepreneurship learning and entrepreneurship ventures

Lately, entrepreneurship and higher education activities have come together to form a new trend of entrepreneurial learning. Entrepreneurs grow and expand by learning, so a thorough theoretical understanding of entrepreneurial learning is critical. On the other hand, entrepreneurial education teaches students to recognize opportunities, seize them, and then use what they've learned to start, manage, and operate their businesses (Zhang et al., 2020). Rive et al. (2017) also stated that entrepreneurial learning is an action that aids in increasing the fundamental knowledge base that is useful in running and initiating new businesses.

Entrepreneurial learning can be thought of as a hands-on activity in which the knowledge gained from an entrepreneur's personal experience is transformed into something that can be used to guide the selection of new skills. However, when looking into the topic of entrepreneurial knowledge, it is necessary to acknowledge that the business experiences of entrepreneurs do not instantly direct the acquisition of entrepreneurial knowledge. In contrast, the acquisition of new practices may then be featured as the growth of new knowledge as a process in which skills are transformed into the knowledge gained through research (Shirish et al., 2021).

For this reason, the learning strategy should focus on encouraging entrepreneurial behavior that emphasizes the development of creativity and critical thinking. This can significantly impact students' ability to grow entrepreneurial skills throughout their careers. Furthermore, these educational endeavors should begin earlier in the educational process than at the end (King and He, 2006). Aside from that, prior studies have shown that entrepreneurial practices and skills include the actual start-up of a new venture and the initial steps that allow a unique venture to begin (Goldsmith and Goldsmith, 2002).

**H2: Entrepreneurial learning has a positive impact on Students' entrepreneurial intentions**

### Role of entrepreneurial learning and education

One of the most popular types of business incubators is the university incubator, which is increasingly being viewed as an engine for inspiring general and local economies by policymakers. This means universities are increasingly being asked to provide capital, faculty time, and effort toward developing new businesses (Hajiha et al., 2014). Some argue that university incubators help new entrepreneurial businesses learn and recognize how to grow through knowledge acquisition, but this isn't necessarily the case (Agudo-Peregrina et al., 2014).

University incubated businesses outperform non-university incubated businesses in sales and employment growth (slope) and sales and employment volume over time (batch) after graduating from the incubator. This is especially true for graduates of universities that have embraced the concept of business incubators (Eskander and Nitschke, 2021). Previous studies demonstrated that entrepreneurial schooling positively impacts entrepreneurs' ability to start and grow new businesses (Ishmuhametov and Kuzmina-Merlino, 2017). Participants in organizations like business incubators appear to offer students exceptional learning opportunities by doing and practicing, proving the importance of social learning and activity-based guidance for practicing thought (Jones and Thornton, 2005).

Reflection of the planned model and the relations between study variables are at the heart of Social Cognitive Theory (SCT). According to this theory, individual characteristics (including cognitions) interact with the environment and behavior. A person's behavior is determined solely by the interaction of these traits (Ramírez-Montoya et al., 2021). Furthermore, the theory emphasizes that an individual's behavior and cognitions directly impact their future behavior (Hauer, 2015). For example, Belton and Stewart (2002) established the following mannequin, which was based on the five collaborative learning (cognitive) areas specific to corporal activity: ecological weather conditions, social, cognitive (i.e., self-efficacy), physiological and personal factors (age and gender) of the individual (i.e., other health behaviors). A person can demonstrate behavior, learn by observation, use self-regulation strategies, predict expected behavior outcomes, and mirror and scrutinize behavior are some of the assumptions of this theory (Jones and Thornton, 2005).

**H3: Students' entrepreneurial education positively impacts students' entrepreneurial intentions**.

As a result of their research (Sareen, 2019), projected entrepreneurial intentions into five distinct categories (1) The basic model of entrepreneurial intention; (2) Personal-level variables; (3) Entrepreneurship education; (4) Institutions and context; (5) the entrepreneurial process. Using Ajzen's theory, we can measure the setting in which entrepreneurship takes place in terms of approach (factors that affect the mind), perceived level of control (contextual factors), and social norms (socio-cultural factors) when it comes to the entrepreneurial act preference, Kim and Yoon's (2021) mode can use two variables to assess an idea's perceived desirability and feasibility.

It is clear that the planned behavior model well-explained process of industrial intent. On the other hand, the relative importance of the various descriptive variables varies depending on the situation.

The following are three hypotheses that we can draw from previous research:

**H4: Students' entrepreneurial intentions are positively influenced by their entrepreneurship attitude**.
**H5: Students' entrepreneurial intentions are influenced by their perceptions of social norms**.

Academic training has a significant influence on future career choices, and this includes the decision of university laureates to pursue a salaried or entrepreneurial career path. Entrepreneurship education programs, even those aimed at learning how to teach students about the concept, should have a positive impact in the short term on their desire to start a business, according to de Kervenoael et al. (2009). This conclusion is supported by a number of empirical studies in various research contexts (Dashti et al., 2019).

According to (Anindito and Handarkho, 2021), an entrepreneurship training program can help raise the entrepreneurial intent of engineering and science students. According to a recent study by Hui-Wen Chuah et al. (2022), entrepreneurship coaching impacts commerce students' entrepreneurial intentions confidently. Instilling in students an important pairing of key functions based on what you've learned, do, and be is an important role of entrepreneurial education in developing future entrepreneurs (Tarekegne and Sidortsov, 2021). According to our research, students trained in entrepreneurship and project management are more likely to become entrepreneurs.

This refers to students' perceptions of what it would be like to start their own business, as stated by Teschner et al. (2020). According to Teschner et al. (2020), Perceptions of students about a person's perception of social norms are shaped by the opinions of influential start-up ideas from their friends and family members. According to Singh et al. (2021), the “degree to which a student believes he can successfully start a new business” is defined as “perceived entrepreneurial capacity.” Education in entrepreneurship is defined as “the entire set of educational and training activities (...) that try to develop in the participants the intention to perform entrepreneurial behaviors, or some of the elements that affect this intention, such as entrepreneurial knowledge, the desirability of the entrepreneurial activity, or its feasibility” (Anand, 2015). “Entrepreneurial intention” refers to the “intentionality among university students to engage in entrepreneurial practices after graduation,” according to Irfan et al. (2021c).

## Research method

### Data collection method and sample

Students at the different Universities in China were asked to fill out a questionnaire. Human resources management and students with a university degree in management strategies were our primary target groups for this study. Students nearing the end of their university studies have completed a 50-h entrepreneurship and project management course.

Faculty and lecturers have long used various teaching methods to introduce students to entrepreneurship, including guest lectures, internships, feasibility plans, field trips, lectures, and case studies (Irfan et al., 2021b). The LHST's entrepreneurial pedagogical program, which adheres to teaching principles, aims to cultivate students' entrepreneurial attitudes, competencies, and abilities (Irfan et al., 2021a). A fictitious entrepreneurial project is used as a vehicle for students to compete against each other in role plays, cooperative learning, case studies, teamwork and simulation. Students who complete this course will be equipped with the knowledge and skills to start their businesses (United Nations Development Programme, 2019).

### Sampling method

We used an empirical sampling method because there was no sampling frame available. As a result, we selected a sample based on sound reasoning (Tangonyire and Akuriba, 2020). After completing the entrepreneurship and project management module, students were asked to fill out a questionnaire. Additionally, data was gathered over the course of a single week in January of this year. More than 98 students from the management program volunteered to participate in this survey (Table 1).

**Table 1:** The demographics of respondents.

**Attributes**	**Characteristic**	**Frequency**	**%**
Age	<19	5	5.1
	19 to 23	67	68.4
	<23	26	26.5
Gender	Male	34	34.7
	Female	64	65.3
Education level	Diploma	45	45.9
	Bachelor	53	54.1
Entrepreneurial ancestry in the family	Yes	15	15.3
	No	83	84.7
Associative experience	Yes	39	39.8
	No	59	60.2
Training wishes	Pseudo-educational project: Learning to teach yourself	57	58.1
	Testimonials from business owners	21	21.4
	Hypothetical course	20	20.4

According to the results, there are 78.1 % females and 42.6 % males in the study sample. At the professional bachelor's, 62.5 % of students studied; at the university diploma of technology level, 34.5 % studied. Over two-thirds (68.4%) of those polled were between 19 and 23 years old. In the survey, 54.08 % of students had already participated in associative activities, while 60.2% never had. 92.7 % of the students revealed that they do not come from a line of business owners. Many of the students who responded to our survey supported the idea of learning by doing (58.1 %).

## Results and discussions

We used Partial Least Squares Path Modeling (PLSPM) to analyze the data measured by the measurement models. In addition, we'll go over the results of our structural model testing.

### Assessing measurement models

The intersecting force indices to be examined are AVE, factor loadings, and composite reliability (CR). After removing nine products with low outer loading values, the Presumed Entrepreneurial Strength statistical method was limited to five items. Convergent validity testing yielded the following results (Table 2).

**Table 2:** Results of converging validity.

**Construct**	**Item**	**Loading**	**Cronbach's alpha**	**Rho-A**	**CR (>0.7)**	**AVE**
Entrepreneurial learning	EL1	0.819	0.917	0.930	0.935	0.764
	EL2	0.824				
	EL3	0.942				
	EL4	0.917				
Perceived Social rule	PSR1	0.807	0.816	0.820	0.903	0.626
	PSR2	0.860				
	PSR3	0.822				
	PSR4	0.770				
Entrepreneurial attitude	EAT1	0.832	0.802	0.838	0.922	0.668
	EAT2	0.778				
	EAT3	0.766				
	EAT4	0.820				
Entrepreneurship education	EED1	0.860	0.899	0.893	0.951	0.595
	EED2	0.873				
	EED3	0.746				
	EED4	0.845				
	EED5	0.824				
Perceived behavior control	PBC1	0.824	0.862	0.866	0.876	0.671
	PBC2	0.837				
	PBC3	0.846				
	PBC4	0.846				
Entrepreneurial Intentions	EINT1	0.909	0.901	0.822	0.835	0.706
	EINT2	0.833				
	EINT3	0.884				
	EINT4	0.915				
	EINT5	0.787				

AVE's Root Square and Cross Loadings are checked to ensure discriminate validity (Al Ghafri et al., 2020). The Truong et al. (2020) criterion can be used to test the discriminant validity of the five latent variables, as shown in the table below (Table 3).

**Table 3:** Discriminate validity results.

**Constructs**	**EL**	**PSR**	**EAT**	**EED**	**PBC**	**EINT**
EL	0.879					
PSR	0.535	0.796				
EAT	0.659	0.627	0.840			
EED	0.592	0.577	0.582	0.793		
PBC	0.592	0.515	0.427	0.529	0.769	
EINT	0.616	0.536	0.444	0.550	0.800	0.582

Furthermore, as evaluated by correlations between constructs, shared between constructs is lower than shared between a construct and its corresponding indicators in terms of variance. For more information, see Table 4.

**Table 4:** Discriminate validity–loading and cross-loading criterion.

**Items**	**Entrepreneurial learning**	**Perceived social rule**	**Entrepreneurial attitude**	**Entrepreneurship education**	**Perceived behavior control**	**Entrepreneurial intentions**
EL1	**0.796**	0.520	0.503	0.462	0.422	0.462
EL2	**0.903**	0.564	0.623	0.537	0.662	0.607
EL3	**0.952**	0.568	0.565	0.501	0.622	0.563
EL4	**0.926**	0.563	0.453	0.435	0.619	0.502
PSR1	0.424	**0.885**	0.530	0.487	0.614	0.544
PSR2	0.509	**0.783**	0.485	0.424	0.387	0.432
PSR3	0.421	**0.835**	0.387	0.444	0.341	0.391
PSR4	0.371	**0.798**	0.241	0.361	0.291	0.298
EAT1	0.561	0.439	**0.878**	0.393	0.315	0.529
EAT2	0.583	0.459	**0.850**	0.466	0.485	0.600
EAT3	0.464	0.504	**0.809**	0.348	0.389	0.515
EAT4	0.436	0.369	**0.765**	0.472	0.435	0.557
EED1	0.449	0.435	0.456	**0.809**	0.460	0.575
EED2	0.483	0.413	0.578	**0.852**	0.575	0.668
EED3	0.514	0.501	0.423	**0.792**	0.548	0.588
EED4	0.438	0.478	0.437	**0.832**	0.559	0.609
EED5	0.337	0.413	0.519	**0.744**	0.443	0.569
PBC1	0.461	0.398	0.465	0.447	**0.821**	0.577
PBC2	0.405	0.327	0.426	0.476	**0.800**	0.568
PBC3	0.570	0.469	0.595	0.553	**0.884**	0.677
PBC4	0.442	0.394	0.461	0.489	**0.814**	0.588
EINT1	0.431	0.385	0.468	0.410	0.421	**0.775**
EINT2	0.618	0.510	0.500	0.495	0.502	**0.836**
EINT3	0.598	0.283	0.536	0.562	0.460	**0.913**
EINT4	0.423	0.397	0.522	0.511	0.543	**0.968**
EINT5	0.550	0.288	0.493	0.411	0.431	**0.888**

The most important information is highlighted in bold.

In conclusion, the measurement model's Validity may be confirmed. For this investigation, we used five models for measuring latent and item factors and a research framework to show the connections between these hypothesized models.

### Assessing structural model

There is a moderate correlation between entrepreneurial intention among management students (R^2^ = 0.621) and the coefficient of determination, indicating that up to 56.1% of the variance can be explained by this endogenous latent construct (Halim et al., 2022). Furthermore, the f2 values multiple epigenetic predictor variables, and attitudes against innovation entrepreneurship training, are within acceptable ranges. On the other hand, a low f2 (f2 = 0.039) index indicates that people do not believe in their entrepreneurial abilities. Perceived social norms do not affect students' entrepreneurial intentions (f2 < 0.02). This study's GoF value (0.584> 0.36) seems to be strong enough to take into account the PLS model's worldwide significance overall (Kumari and Bhateja, 2022). Figure 2 shows the model's predictive power, which is acceptable (Q2 = 0.348), as can be seen.

**Figure 2:** Structural model analysis results. *** significance at 1%.

Students' entrepreneurial intentions are largely influenced by their education and attitude toward entrepreneurship. This shows that the relationship between students' entrepreneurial intentions and perceptions of social norms and their perceived entrepreneurial capacity is insignificant (Table 5).

**Table 5:** Result of hypothesis testing.

**Hypothesis**	**Path**	**β-value**	**t-value**	**p-value**	**Decision**
H1	EL → EINT	0.468***	3.111	0.001	Supported
H2	PSR → EINT	0.149	0.968	0.379	Not supported
H3	EAT → EINT	0.131***	1.900	0.004	Not supported
H4	EED → EINT	0.380***	3.267	0.003	Supported
H5	PBC → EINT	0.290***	2.311	0.002	Supported

*** significance at 1%.

As presented in Table 5, the findings shows that entrepreneurial learning has a significant and positive influence on management students' entrepreneurial intentions. The findings made it possible to accept this hypothesis (EL → EINT: H1. β = 0.468; *t* = 3.111; p = 0.001). Moreover, there is an insignificant association between perceived social rules and management students' entrepreneurial intention (PSR → EINT: H2, β = 0.131, *t* = 0.968 and *p* = 0.379). A student's attitude toward entrepreneurial activity accounts for 13.1% of the explanation of their intended entrepreneurial behavior. In addition, entrepreneurship education (EED → EINT: β = 0.380^***^; *t* = 3.267; *p* = 0.003) and perceived behavior control (PBC → EINT: β = 0.290^***^; *t* = 2.311; *p* = 0.002) have a significant positive impact on management students' entrepreneurial intention. Findings from a TPB-based study were used to identify variables that could impact students' entrepreneurial intentions and question entrepreneurship education's role. The data shows that various factors influence students' entrepreneurial intentions.

### Conclusion and policy recommendation

Our research shows that management Students' attitudes toward entrepreneurship influence their entrepreneurial intentions. The TPB is linked to this correlation in numerous studies (Tanveer et al., 2021). Entrepreneurial research has yielded a number of empirical findings that attitudes toward the entrepreneurial act are a significant determinant of the individual's entrepreneurial intention (Ai et al., 2022). based on an empirical study involving 97 former students of a business school, students' intentions toward entrepreneurship can be explained by their perception of feasibility and attitude toward action. According to Lăzăroiu et al. (2020), who studied 94 students who had just graduated from the Sfax higher business school, attitudes about behavior and social norms influence whether or not students want to start their own business. A study of 250 university students by Jiménez et al. (2021) found a similar positive correlation. It was found that students' attitudes toward entrepreneurship have an impact on their entrepreneurial intentions (Campbell, 2019). Furthermore, in the Chinese context, authorities and universities can play a significant role in improving the intention level of university students to start a business.

According to the findings, social norms cannot predict students' entrepreneurial intentions. In line with the findings of Astawa et al. (2021), these results show no discernible impact on students' entrepreneurial intentions from this variable. Furthermore, Venkatesh and Davis (2000) show that students' entrepreneurial intent to start a new business is unaffected by social recognition in Portugal and Brazil. Many previous studies have suggested that students' perceptions of social or subjective norms can influence their entrepreneurial intentions. On the other hand, the Chinese do not recognize or value student entrepreneurship.

In light of the empirical evidence, we can conclude that students' entrepreneurial intentions are not affected by their perceptions of entrepreneurial capability. The lack of self-confidence and low self-esteem among management students in Chinese HEIs could explain this finding.

According to previous empirical studies, students' entrepreneurial intentions are positively influenced by their entrepreneurial capacity (Hamari, 2013). For example, a study of 245 undergraduates found that students' intentions to start a new business were better explained by their belief in their entrepreneurial self-efficacy. Studying business students from public universities, Kolotylo-Kulkarni et al. (2021) also found a connection between the two variables.

According to the findings of this study, students' entrepreneurial intentions can be explained by the rank of entrepreneurship education. As a result, entrepreneurship education is vital for developing students' entrepreneurial aspirations. A learning-by-doing approach to entrepreneurial training benefited the students who took part in our research. Using this teaching method, students' entrepreneurial intentions and behavior are fostered and improved by teachers having direct contact with their students. Additionally, entrepreneurship education influences students' entrepreneurial inspiration and helps improve their entrepreneurial mindset through propensity, tolerance, risk, ambiguity and the ability to recognize and seize opportunities.

Studies show that students' plans to start their own business are better explained when they receive entrepreneurship training. Several other studies have almost confirmed the Validity of these findings. Education programs and training courses have been shown to raise students' entrepreneurial intentions, according to an empirical study involving 374 Norwegian students (Lu et al., 2012). Similarly, among French students, Burton-Jones and Hubona (2006) found that entrepreneurship training has a positive and significant effect on their entrepreneurial intentions. An investigation by Dubey, involving 276 students from 34 countries, found that entrepreneurship training provides entrepreneurial skills and makes the growth of their entrepreneurial intentions more conductive. According to the research, the three dimensions of entrepreneurial orientation–proactiveness, innovation, and risk-taking–can be explained by entrepreneurship training. Recently, a study by Baron and Kenny (1986) found that educating students about entrepreneurship increases their likelihood of starting their own business in the near future. But some empirical studies have shown that an entrepreneurial education program has a negative relationship with the intention to become an entrepreneur.

### Theoretical and practical implications

The entrepreneurial aspirations of management students could now be predicted using a simplified model developed in the current study. According to the study's findings, students at Chinese higher education institutions have strong entrepreneurial intentions. Identifying the factors influencing students' entrepreneurial intentions is critical to developing policies and training programs that encourage entrepreneurial behavior among university students. This study's findings have theoretical implications and practical recommendations for universities, business school instructors, and public officials.

Students' entrepreneurial intentions can be better understood by understanding their entrepreneurial education. As a result of this research, a new understanding of management students' entrepreneurial intentions is developed. The present study contributes to the literature on entrepreneurship education by looking at entrepreneurship education in HEIs using learning by doing pedagogy. The findings of this study have theoretical implications.

This study has limitations due to the small sample size and a limited number of variables used to predict entrepreneurial intentions. Theory-based prediction of management students' entrepreneurial intentions is another theoretical contribution. In addition to entrepreneurship, we are extending TPB's use to entrepreneurship education. According to our study, students' intentions to start a new business are positively influenced by their attitude toward entrepreneurship and entrepreneurial education. Entrepreneurship education can serve as a stepping stone for future entrepreneurs. According to research on participation in entrepreneurship education programs, entrepreneurial self-efficiency, life transitions, desirability, entrepreneurial intent, barriers and opportunities, and information and resources are all important regulating variables. Researchers identified these six variables. Students in the sports industry could also benefit from an entrepreneurial learning method (Ashraf et al., 2021b). As we've found in previous studies, students' entrepreneurial intentions can be bolstered through a curriculum that emphasizes hands-on activities like business plan development simulations and group discussions.

This study's findings show that students' entrepreneurial intentions and activities can be strengthened by incorporating entrepreneurship education into their curricula from a practical standpoint. According to the study, universities in China need to incorporate entrepreneurship education programs into their curriculums.

Results like these motivate us to dig deeper into entrepreneurship education methodologies and their long-term effects on entrepreneurial intents and behaviors toward business creation. There are two distinct but intertwined roles that the Chinese Higher Education Institutions (HEIs) must fulfill. For starters, the delivery of an entrepreneurship training program that aims to increase students' entrepreneurial aspirations. The second goal is to assist students in developing innovative business ideas by establishing academic incubators for innovation and entrepreneurship.

More and more people agree that collaborating with the entrepreneurial ecosystem, including entrepreneurs, businesses, financial institutes, incubators and accelerators, governments and non-profits, is critical to the success of entrepreneurship education programs (Cenfetelli et al., 2005; Bolaños et al., 2022). As a result, Chinese higher education organizations are encouraged to participate in this collaborative effort. In the same way, stakeholder engagement is essential to the success of entrepreneurship education.

The development of three complementary capabilities should focus on entrepreneurship training: attitude (ambiguity acceptance, self-efficiency), skills, and self-insight (financial and marketing). In entrepreneurship education, teachers play a critical role. Teachers must provide a learning-by-doing approach based on action learning that integrates theory with practical applications in academic entrepreneurship education (Davis and Lang, 2012). Guest speakers, business game business, group discussions, simulation case studies and plan development are examples of activist teaching methods that can encourage entrepreneurial behavior among management students (Jinru et al., 2021).

Chinese universities must implement methods and e-learning systems to incorporate education across time and space. According to Malesios et al. (2021) and colleagues, e-learning can help students develop entrepreneurial skills and competencies. An online entrepreneurship program allows students to take courses at their convenience, regardless of their distance from the university.

As a result of our research, we also offer concrete policy recommendations. As a tactical tool for local growth, entrepreneurship education and training programs in developing countries like China can help boost entrepreneurial activity, creating new businesses and jobs (Merabet et al., 2021). Representatives in China are invited to develop public policies promoting entrepreneurial education programs, including various regional investors, such as support structures, qualified mentors, the chambers of business, services and industry; the ProSource foundation and the general confederation of Chinese enterprises.

### Limitations and future research

This study has limitations due to the small sample size and a limited number of variables used to predict entrepreneurial intentions. A larger sample of Chinese universities can be used in future research to predict the entrepreneurial intent of management students better. The role of socio-cultural background, personal characteristics, and emotional intelligence in predicting the entrepreneurial intentions of management students would also be interesting to investigate.

Further empirical studies are needed to understand how entrepreneurship education can encourage students in other fields, such as sports or engineering. Additionally, more research into how digital academic entrepreneurship affects student motivation and behavior to start their own business is warranted.

## Data availability statement

The raw data supporting the conclusions of this article will be made available by the authors, without undue reservation.

## Author contributions

Both authors listed have made a substantial, direct, and intellectual contribution to the work and approved it for publication.

## Conflict of interest

The authors declare that the research was conducted in the absence of any commercial or financial relationships that could be construed as a potential conflict of interest.

## Publisher's note

All claims expressed in this article are solely those of the authors and do not necessarily represent those of their affiliated organizations, or those of the publisher, the editors and the reviewers. Any product that may be evaluated in this article, or claim that may be made by its manufacturer, is not guaranteed or endorsed by the publisher.
